# Prediction of Hearing Prognosis of Large Vestibular Aqueduct Syndrome Based on the PyTorch Deep Learning Model

**DOI:** 10.1155/2022/4814577

**Published:** 2022-04-13

**Authors:** Bo Duan, Zhengmin Xu, Lili Pan, Wenxia Chen, Zhongwei Qiao

**Affiliations:** ^1^Department of Otolaryngology-Head and Neck Surgery, Children's Hospital of Fudan University, Shanghai 201102, China; ^2^Department of Radiology, Children's Hospital of Fudan University, Shanghai 201102, China

## Abstract

In order to compare magnetic resonance imaging (MRI) findings of patients with large vestibular aqueduct syndrome (LVAS) in the stable hearing loss (HL) group and the fluctuating HL group, this paper provides reference for clinicians' early intervention. From January 2001 to January 2016, patients with hearing impairment diagnosed as LVAS in infancy in the Department of Otorhinolaryngology, Head and Neck Surgery, Children's Hospital of Fudan University were collected and divided into the stable HL group (*n* = 29) and the fluctuating HL group (*n* = 30). MRI images at initial diagnosis were collected, and various deep learning neural network training models were established based on PyTorch to classify and predict the two series. Vgg16_bn, vgg19_bn, and ResNet18, convolutional neural networks (CNNs) with fewer layers, had favorable effects for model building, with accs of 0.9, 0.8, and 0.85, respectively. ResNet50, a CNN with multiple layers and an acc of 0.54, had relatively poor effects. The GoogLeNet-trained model performed best, with an acc of 0.98. We conclude that deep learning-based radiomics can assist doctors in accurately predicting LVAS patients to classify them into either fluctuating or stable HL types and adopt differentiated treatment methods.

## 1. Introduction

Large vestibular aqueduct syndrome (LVAS), also known as congenital enlarged vestibular aqueduct, is a congenital inner ear malformation with a high clinical incidence [1]. The disease is mainly caused by malformations or containment of ductus endolymphaticus, with sensorineural deafness, tinnitus, and other hearing disorders as well as dizziness and balance disorders as the main clinical manifestations, seriously affecting children's health. The mechanism of hearing loss (HL) in LVAS patients remains uncharacterized [2]. Although without an effective treatment, the wide application of high-resolution computerized tomography (CT) and magnetic resonance imaging (MRI) has improved the diagnosis rate of this disease in recent years, providing an important basis for clinical research of this disease. Hearing aids are recommended for patients with residual hearing, while for those with extremely severe deafness, cochlear implants are indicated. Whereas, there is currently no consensus on whether patients with residual hearing should be treated with cochlear implants or hearing aids. Generally speaking, most LVAS patients will experience hearing fluctuations, stepwise HL, and even extreme deafness, while only a few have stable hearing [3]. Therefore, it is particularly important to screen out patients with stable hearing in the early stage to avoid overtreatment and to identify those with more hearing fluctuations and poor treatment effects to guide close follow-ups.

The concept of radiomics was first proposed by Dutch scholars [4] in 2012, which emphasizes the deep meaning of high-throughput extraction of a large amount of image information from images (MRI, CT, positron emission tomography [PET], etc.) to achieve tumor feature extraction, segmentation, and model building and assist clinicians to make more accurate diagnosis through in-depth analysis, mining, and prediction of a large amount of image data information. Radiomics can be simply interpreted as transforming visual image information into deep features for quantitative research [5]. In recent years, the organic integration of medical image-aided diagnosis and big data technology has produced a new radiomics methodology, which can extract a large number of features from images to quantify tumors and other major diseases and help effectively solve the problem that tumor heterogeneity is difficult to quantitatively evaluate, with huge clinical implications. The radiomics technology is derived from computer-aided diagnosis (CAD) and has developed into a method of auxiliary diagnosis, prediction, and analysis of clinical, image fusion, genetic, and other information. With the proposal of this new research method, more and more researchers are trying to comprehensively evaluate various tumor phenotypes by using the data extracted from radiomics [6]. The imaging feature analysis by radiomics in otolaryngology and head and neck surgery is relatively rare, and this paper, as far as we are aware, is the first to study its application in the structural characteristics of the endolymphatic sac. This paper is a retrospective analysis aiming to explore the application value of the artificial intelligence (AI) model of internal acoustic meatus (IAM) magnetic resonance (MR) in predicting hearing fluctuations, as well as to predict the hearing prognosis of LVAS patients by radiomics.

## 2. General Information and Proposed Methods

### 2.1. General Information

Patients with hearing impairment were collected from the Department of Otolaryngology, Head and Neck Surgery, Children's Hospital of Fudan University from January 2001 to January 2016. After the early diagnosis of deafness, patients were diagnosed as LVAS by IAM MR examination and had been followed up in our hospital for at least 4 years. Deafness caused by autoimmune diseases and other diseases were excluded. Definition of hearing fluctuation: patients whose pure tone average (PTA) showed an overall change in HL of less than 10 dB from the initial to the last audiogram were considered to have stable HL. Those with HL PTA greater than or equal to 10 dB from the initial to the latest HL were considered as progressive HL with fluctuations. We used the HL PTA threshold of 70 dB to define cochlear implant candidacy or severe HL. In this part of the analysis, patients with initial PTA greater than 70dB HL were excluded [7]. The follow-up was conducted by means of game audiometry or brainstem evoked potential or pure tone audiometry, and the interval was usually 3 months. Patients received timely outpatient treatment in the case of hearing fluctuations. The hearing was followed up for at least 4 years. Children with unilateral LVAS were excluded, as well as those with unilateral hearing fluctuations.

This study screened out the eligible cases, with a total of 59 children enrolled. Among them, there were 30 cases of bilateral hearing fluctuation accompanied by HL, with poor treatment effects. The rest 29 children were with stable bilateral hearing; the number of HL was less than 2 times in 4 years, with the hearing basically recovered to the original level after effective drug treatment and the final HL no more than 10 dB.

### 2.2. Proposed Methods

The processing flow of radiomics is summarized as follows:

1. Step 1: acquisition of image data and collection of original IAM MR data in a DICOM format
2. Step 2: selection of the layers containing the cochlea, vestibule, semicircular canal, ductus endolymphaticus, and inner lymphatic sac, as can be seen in Figure 1
3. Step 3: LabelMe software is applied to label the regions of interest (ROIs) of patients' MR images. The image database is established; there were 46 images in the fluctuating HL group and 443 in the stable HL group
4. Step 4: deep learning classification and prediction. *Python* was used to build deep learning convolutional neural networks (CNNs) with the learning rate of 0.01 and the training epoch of 200. Later, VGG, GoogLeNet, and ResNet networks were used for classification and prediction. Accuracy, specificity, sensitivity, and area under the curve (AUC) can be used to evaluate the performance of the classifiers [8].

## 3. Results and Discussion

The confusion matrices of VGG16, VGG19, ResNet18, ResNet50, and GoogLeNet are shown in Tables 1 and 2.  Figure 2 shows the areas under the receiver operating characteristic (ROC) curves. Vgg16_bn and vgg19_bn, CNNs with fewer layers, yield better effects. ResNet18 and ResNet50, CNNs with more layers, have relatively poor effects. The GoogLeNet-trained model performs best. Theoretically, the PTA threshold for HL of cochlear implant candidates is approximately 70 dB, but for LVAS patients with stable hearing, the therapeutic effect of hearing aids is not worse than that of cochlear implants. It is important to distinguish LVAS patients with stable hearing.

In addition, vgg16_bn, vgg19_bn, and ResNet18, convolutional neural networks (CNNs) with fewer layers, had favorable effects for model building, with accs of 0.9, 0.8, and 0.85, respectively. ResNet50, a CNN with multiple layers and an acc of 0.54, had relatively poor effects. The GoogLeNet-trained model performed best, with an acc of 0.98. We conclude that deep learning-based radiomics can assist doctors in accurately predicting LVAS patients to classify them into either fluctuating or stable HL types and adopt differentiated treatment methods.

## 4. Discussion

In terms of exploring the CT and MRI features of LVAS patients, as well as the relationship between MRI classification of the endolymphatic sac and the degree of HL, most studies focus on the diameter of the bony opening of the vestibular aqueduct and the volume of the endolymphatic sac. Their conclusions are mainly that the degree of HL in patients with LVAS had no significant correlation with the diameter of vestibular aqueduct orifice and the signal changes of the endolymphatic sac. There is a lot of basic research on the mechanism of deafness, including SLC26A4 gene and animal models [9], but it does not help much in predicting the prognosis of hearing. In previous studies, radiomics and AI have mostly focused on tumor research. AI has made remarkable progress in recent years. The development of multilayer network architectures, which can compile mathematical functions with millions of parameters, enables machines to think deeply and interpret complex data in a highly precise manner. Radiomics is the result of AI application in the field of medical imaging, which can indirectly reflect the microscopic changes of genes or proteins of tissues at the macroscopic level. The purpose of this study is to develop a machine learning model based on IAM MR of patients to predict hearing fluctuations.

Mey et al. discussed the relationship between the single allele (M1), double allele (M2), and mutation deletion (M0) of the SLC26A4 gene and the morphology and hearing level of the inner ear and found that the number of SLC26A4 mutations was associated with the severity and variability of inner ear morphology and the hearing level in patients with LVAS. The hearing of M2 individuals is poor, the cochlea type II is mainly incomplete, and the endolymphatic sac is enlarged. As for M1 individuals and those without SLC26A4 mutation, the HL is less, and the inner ear morphology is more diversified. However, they fail to predict the hearing prognosis of patients well.

VGG [10]: VGG16 replaces the large kernel-sized filters (11 × 11, 7 × 7, and 5 × 5) in AlexNet with several 3 × 3 kernel-sized filters one after the other. For a given receptive field (the local size of the input picture related to the output), using stacked small convolution kernels is superior to using large convolution kernels, because multilayer nonlinear layers can increase the network depth to ensure the learning of more complex patterns, with relatively lower cost (fewer parameters).

GoogLeNet [11]: Inception (also called GoogLeNet) is a brand new deep learning structure proposed by Christian Szegedy in 2014. Prior to this, structures such as AlexNet and VGG all achieved favorable training effects by increasing the depth (number of layers) of the network, but the increase in the layer number would bring many negative effects, such as overfit, gradient disappearance, and gradient explosion. Inception is proposed to improve the training results from another perspective: it can make more efficient use of computing resources and extract more features with the same amount of computation, thus improving the training results.

ResNet [12]: ResNet, which was proposed in 2015 by researchers at Microsoft Research, introduced a new architecture called residual network. ResNet won the championship in the ILS VRC (ImageNet Large Scale Visual Recognition Challenge) in 2015. Its main contribution is the discovery of “Degradation” and the invention of “Shortcut connection” in response to the degradation phenomenon, which greatly eliminates the difficulty of neural network training with too much depth.

Vgg16_bn and vgg19_bn, CNNs with fewer layers, can produce better effects [13, 14]. ResNet18 and ResNet50, CNNs with more layers, do not have such favorable effects [15]. GoogLeNet-trained models worked best, with 98 percent accuracy. In LVAS, the area of the target organ's lymphatic sac and the cochlea accounts for a small proportion of the whole picture. While in fact, the more layers of the neural network, the larger the deep receptive field, so it is not suitable for case studies of small lesions. Deep learning generally requires a large amount of data, perhaps millions of images to produce a good model effect. However, it is difficult to accumulate data of this magnitude in medicine, which usually can only collect thousands of pictures, let alone rare diseases. Transfer learning is a machine learning method that transfers knowledge from one domain (i.e., source domain) to another domain (i.e., target domain) so that the target domain can achieve better learning effects [16]. There is no need to recollect and calibrate huge new data sets at great cost, or the data may not be available at all. For the rapidly emerging new fields, this learning method can quickly migrate and apply them, reflecting the advantages of timeliness. So, transfer learning can be considered if the training model of deep learning is not effective [17]. Other well-trained models with better effects can be migrated, such as ImageNet classification of cats and dogs, or some better models trained by yourself. In this way, the data demand for this training can be significantly reduced, and the effect will be significantly improved.

The image features of deep learning are highly dimensional with no physical meaning, so there is no way to discuss their physiological meaning for the time being. Therefore, the deep learning model of this study can only be used for classification temporarily and may be used for 3D separation in further research.

While understanding the correlation between deafness and MR in LVAS patients, another goal of this work is to establish an interpretable medical application system. In the medical field, the number of data sets will never be as large as the current benchmark databases, such as ImageNet [18], which has more than millions of images. Therefore, a system that uses a limited number of data sets while still achieving good performance will have a major impact on medical applications.

The use of radiomics feature analysis can avoid multiple imaging examinations, and even the diagnosis of lesions can be confirmed by the analysis of imaging features with the images of a single imaging examination [19]. Texture analysis is one of the feature data of radiomics, a system gradually realized through segmentation of lesions, feature data extraction, database establishment, and analysis of individualized data. Through the research of radiomics and texture analysis, we can decode the huge amounts of digital information hidden in medical images and objectively apply it to the clinical diagnosis and treatment of diseases and the analysis of prognosis [20].

Texture analysis and radiomics have been widely applied in various systems of neoplastic lesions in recent years due to their objective and descriptive characteristics [21]. Among them, the phenotype of tumors can be evaluated in depth and objectively based on the heterogeneity of tumors, providing accurate guidance for differential diagnosis, treatment, and prognosis prediction of tumors. However, there are still some technical problems, such as image acquisition mode, reconstruction parameters, tumor size, and segmentation threshold, which will affect the feature results. Some texture features also have the limitation of poor repeatability [22, 23]. With regard to image segmentation, manual image segmentation will result in interobserver differences, so automatic or semiautomatic image segmentation is usually recommended. As for feature calculation, there are also different calculation methods for the same texture feature. At present, scholars pay little attention to their application in nonneoplastic diseases [24]. Given their certain potential and value for the research of nonneoplastic diseases in various systems, finding feasible means to select the most stable and optimal texture features from a large number of texture features is the focus and difficulty of current research.

## 5. Conclusions

We conclude that radiomics based on deep learning can assist doctors to accurately predict LVAS patients and classify them into hearing fluctuation type and hearing stability type. For patients with stable hearing, conservative treatment is recommended if hearing aid therapy can meet life needs. While for those with hearing fluctuations, close follow-ups or cochlear implant surgery is indicated.

There are some deficiencies in this study that need to be addressed. First, the number of cases enrolled is limited, so it is necessary to expand the sample size for further study to improve diagnostic accuracy. Second, patients with unilateral LVAS and those with unilateral hearing fluctuation of bilateral LVAS were excluded. Due to the small sample size, it is not suitable for deep learning research. So, more cases with different types should be collected to expand the sample size for further research. Third, the MR data of this study were all from the same MR scanning instrument in our hospital, without data from other hospitals for verification. The MR data were all T2 sequences with a layer thickness of 1 mm, while images of other layer thicknesses have not been studied. Therefore, the robustness of the model needs to be further determined. In future studies, we can combine the gene, temporal bone CT, and MR of other sequences to conduct modal studies, so that the feature information will be more sufficient. Last but not the least, 3D separation of the endolymphatic sac, vestibule, and cochlea, as well as surrounding brain tissue can also be carried out for 3D model research, which may be more in line with the real world.

The radiomics feature analysis based on deep learning can be used as an important auxiliary means to differentiate and diagnose LVAS hearing as stable or fluctuating, which can provide important clues for early noninvasive diagnosis, guide further clinical treatment, and avoid great interference to children's language, understanding, and learning abilities caused by delayed treatment.

## Figures and Tables

**Figure 1:** The red arrows indicate the bilateral inner ear and the endolymphatic sac, in which the endolymphatic sac includes high- and low-signal intensity areas.

**Figure 2:** Areas under the receiver operating characteristic (ROC) curves.

**Table 1:** The accuracy, precision, recall and F1-score of VGG16, VGG19, ResNet18, and ResNet50.

vgg16_bn		vgg19_bn		ResNet18		ResNet50		GoogLeNet	
85	8	66	27	78	15	22	71	91	2
9	84	9	84	12	81	14	79	4	89

**Table 2:** The accuracy, precision, recall and F1-score of different models.

	acc	Recall	Precision	f1_score
vgg16_bn	0.9	0.9	0.91	0.91
vgg19_bn	0.8	0.9	0.75	0.82
ResNet18	0.85	0.87	0.84	0.85
ResNet50	0.54	0.85	0.52	0.65
GoogLeNet	0.98	0.96	0.98	0.97

## Data Availability

The simulation experiment data used to support the findings of this study are available from the corresponding author upon request.
